# Experimental Study on Properties of Methane Diffusion of Coal Block under Triaxial Compressive Stress

**DOI:** 10.1155/2014/385039

**Published:** 2014-11-03

**Authors:** Hong-Bao Zhao

**Affiliations:** ^1^College of Resources and Safety Engineering, China University of Mining and Technology (Beijing), Beijing 100083, China; ^2^State Key Laboratory of Oil and Methane Reservoir Geology and Exploitation (Southwest Petroleum University), Chengdu 610500, China; ^3^State Key Laboratory of Coal Resources and Safe Mining, China University of Mining & Technology, Beijing 100083, China

## Abstract

Taking the standard size coal block samples defined by ISRM as research objects, both properties of methane diffusion of coal block under triaxial compressive stress and characteristic influences caused by methane pressure were systematically studied with thermo-fluid-solid coupling with triaxial servocontrolled seepage equipment of methane-containing coal. The result shows the methane diffusion property of coal block under triaxial compressive stress was shown in four-stage as follow, first is sharply reduce stage, second is hyperbolic reduce stage, third is close to a fixed value stage, fourth stage is 0. There is a special point making the reduced rate of characteristic curve of methane diffusion speed become sharply small; the influences of shape of methane diffusion speed characteristic curve caused by methane pressure are not obvious, which only is shown in numerical size of methane diffusion speed. Test time was extended required by appear of the special point makes the reduce rate of methane diffusion speed become sharply small. The fitting four-phase relation of methane diffusion of coal block under triaxial compressive stress was obtained, and the idea is proposed that influences of the fitting four-phase relation caused by methane pressure were only shown in value of fitting parameters.

## 1. Introduction

Most of coal or weak rock is in triaxial stress state near stope of underground coal mining; triaxial stress state apparently has influences on the internal structure of coal or weak rock, and internal structure is the main storage and transport place in coal block. All of these will make the storage and transport characteristics of methane in coal or weak rock be changed because of influences on the internal structure of coal or weak rock. Power of methane flow is methane pressure gradient, which is determined by the change of methane desorption or adsorption caused by the change of stress state in coal or weak rock. And lots of methane stored in coal mass ahead of mining work face, if the coal mass was continued mining, stored methane will be desorbed so that the methane pressure gradient will formed in the coal mass, which will make methane constantly migration to the coal wall and gush into the extractive space at last.

The majority of studies [1, 2] on this research area concentrated on methane diffusion law of pulverized coal and the methane diffusion law of mining work face by scholars abroad and in China. For example, the methane diffusion characteristics of tectonic coal were studied by Fu et al. [3], and the differences of methane diffusion characteristics between tectonic coal and nontectonic coal were obtained. The mathematical model and the numerical solver on methane diffusion of coal particles were studied by Qin et al. [4]; the measured curves of different particle diameter between accumulated desorption amount and test time were obtained in different initial pressure. The methane diffusion characteristics of coal block were studied by Li et al. [5]; the differences of methane diffusion characteristics between coal block and coal particles were obtained. The methane diffusion characteristics of coal mass affected by acoustic field were studied by Li et al. [6]; the influence law of methane diffusion characteristics of coal mass caused by acoustic field was obtained. The methane diffusion characteristics of coal containing water were studied by Mou et al. [7]; the influence law of methane diffusion characteristics of coal mass caused by injected water was obtained, and so forth. Although many research works [8–10] have been done and fruitful results have been obtained, there are the following issues, for example, taking pulverized coal as the research object, but the influence of the internal structure of coal mass is not considered, and the free state of coal is taken as research environment, but the influence caused by stress state is not considered. But the internal structure of coal block has critical influences on the storage and transport characteristics of methane, and the stress state of coal block also has critical influences on the change of internal structure of coal block. Therefore, the methane diffusion law will be studied by systematic experiment when the coal block is in triaxial stress state in this paper.

## 2. Test Equipment and Test Programs

### 2.1. Test Equipment

All tests of this paper were done in State Key Laboratory of Coal Mine Disaster Dynamics and Control belonging to Chongqing University. Thermo-fluid-solid coupling with triaxial servocontrolled seepage equipment of methane-containing coal was the key equipment when tests of this paper were done in the laboratory, which is shown in Figure 1. The main technical parameters of the equipment include that the available maximum axial stress is 100.0 MPa, the available maximum confining stress is 10.0 MPa, and the available maximum methane pressure is 6.0 MPa, whose accuracy of stress value is ±0.5% and the accuracy of strain value is ±0.1%; the system of data acquisition consists of ring extensometer produced by Epsilon in America and methane mass flow controller produced by Beijing Sevenstar Electronics Co, LTD. The equipment automatically collects data including stress, strain, temperature, and amount of methane mass flow. All of the mechanics tests of coal block containing methane, penetration properties tests of coal block, and desorption or adsorption characteristic tests can be done by the equipment very well.

### 2.2. Test Programs

The briquette samples made by crushed raw coal collected from the mining work face were taken as research objects; the diffusion characteristics of methane when methane pressure is not fixed are studied under fixed triaxial compressive stress state. When the tests were done, the axial stress is fixed in 5.0 MPa and confining pressure is 6.0 MPa, but the methane pressure is changed among 1.0 MPa, 2.0 MPa, and 3.0 MPa (according to gas pressure of work face of mine, and appropriately sized gas pressure gradient is considered, too). Before tests were done, the stress including axial stress and confining pressure was alternately raised until reaching the designed value, and the fixed pressure methane was exerted lasting 24 hours in order to make the coal block adsorbed methane diffuse fully. The fixed pressure methane will be stopped and the control valve was opened in order to make the methane contained in coal block diffusion gush freely from coal block; the properties of methane diffusion speed were monitored from time to time. The tests of every fixed methane pressure level are done from three to five times according to the law of ISRM. The samples used by tests were shown in Figure 2.

## 3. Results and Analysis of Tests

### 3.1. Tests of Methane Diffusion Properties

According to the designed test program, the smallest unit of mass flow controller is taken as mark of end of methane diffusion test, and characteristics curve of methane diffusion test was divided into two parts taking 1.0 L/min for the boundary in order to get comparable law (the methane diffusion speed of coal block at the beginning of curves is much larger than its size at the later stage; 1.0 L/min is taken as dividing point). The characteristics curve of methane diffusion speed of coal block under fixed triaxial compressive stress state was shown in Figure 3.

According to the analysis in Figure 3, the following can be obtained.

(1) The characteristics curve of methane diffusion speed of coal block under fixed triaxial compressive stress state can be divided into four stages, including first is sharply reduce stage, second is hyperbolic reduce stage, third is close to a fixed value stage, fourth stage is 0. Among the four stages, the stage of approaching a small fixed value is the longest part in process of test time.

(2) At the beginning of methane diffusion test of coal block under fixed triaxial compressive stress state, the methane diffusion speed is large and the rate of reduction is large, too. The reason may be that there is some high pressure methane in test system piping and it will gush out at once lasting a period after the control valve is opened. Although it also includes methane diffusion of coal block, the amount of methane diffusion is much smaller than methane emission from test system piping.

(3) Apparent style of hyperbolic curve is shown and there is a special point which makes the curve appear rapid change after the methane diffusion test of coal block under fixed triaxial compressive stress state enters the second stage. The reason may be that the amount of methane diffusion of coal block has occupied the main part as methane diffusion completely fully in test system piping, because partial free methane is contained in coal block and the methane pressure is much bigger, which makes the amount of free methane transformed from absorbed methane also larger and larger, so that the methane diffusion speed is larger and the rate of reduction is larger and lasting time is short. When the free methane diffusion is completed, the methane pressure will gradually decrease at the same time, so that methane diffusion speed is small and the reduction rate of methane diffusion speed is decreased, which is shown, too.

(4) All properties of small methane diffusion speed, small reduction rate, and lasting long time were shown in fixed triaxial compressive stress state after the test curve enters the third stage. The reason may be that the emission of methane only consists of free methane that is changed from adsorbed methane in coal block after the initial free methane is diffused completely so that the methane diffusion speed is small. Because the methane pressure will decrease gradually at this stage, the time needed by free methane changed from absorbed methane became longer and longer, which will also last a long time. Additionally, the compress effect on pore and crack structure in coal block caused by triaxial compress stress will become more and more obvious as the diffusion of methane in coal block, which makes the methane flow channel become narrow so that the methane flow becomes more and more difficult; all of these are main reasons that caused the law to be shown.

(5) Curve of methane diffusion speed of coal block under fixed triaxial compress stress state shows that methane diffusion speed will come to the value of 0 finally, but it needs a very long time. The reason may be that free methane has been gradually diffused completely in coal block as the extent of test time, and most of absorbed methane has been transformed into free methane and diffused out, and residual methane in coal block will be diffused out completely as the extent of test time; all of them are the main reasons for the law.

(6) The first stage and the third stage of the curve of methane diffusion speed of coal block under fixed triaxial compress stress state can be expressed by approximate linear relationship, but the second stage is expressed by hyperbolic. The differences between obtained law from coal block in triaxial compress stress state and pulverized coal in free state are the size of obtained fitting equation parameters.

(7) The law obtained from laboratory tests is similar to the law obtained from mining work face; the common law is that the amount of methane diffusion is large at the beginning of the coal wall exposure, and the amount of methane diffusion will come to the value of 0 finally as the extent of exposed time.

(8) The results obtained from tests not only are used to analyze source and composition of diffusion methane, but also can be used to show the fact that the briquette specimens can be used to test instead of raw coal; the difference of obtained law will only be shown in the size of parameters.

### 3.2. Study on the Influence of Methane Diffusion Properties Caused by Methane Pressure

Methane pressure in coal block is formed by free methane; the size of methane pressure not only can be used to show the amount of methane in coal block, but also has a direct impact on methane diffusion speed of coal block. In order to get the influences on methane diffusion speed properties of coal block under triaxial compressive stress caused by methane pressure, the curves of methane diffusion speed of coal block under triaxial compress stress were studied in the different methane pressure according to the designed test program on level of 1.0 MPa, 2.0 MPa, and 3.0 MPa, shown in Figure 4 (because the differences are small among these curves, if these curves are drawn in a common figure, the differences will not be noticed, so they are dealt with as in Figure 4).

According to the analysis in Figure 4, the following can be obtained.

(1) Influences caused by methane pressure on curves of methane diffusion speed of coal block under triaxial compress stress are not obvious; the four-stage property of the curve is still very obvious as the methane pressure is raised or decreased.
(2) Obvious influences are shown in part of the size of methane diffusion speed because of different methane pressure. The lasting time of large methane diffusion speed is extended and the reduction rate of methane diffusion speed is reduced with the raising of methane pressure at the same time. The reason may be that the amount of methane remaining in test system piping is raised and the amount of free methane in coal block is much larger with the increase of methane pressure; all of them will cause the law.
(3) Special point that makes the reduction rate of methane diffusion speed of coal block sharply reduce will appear after a long test time with the increase of methane pressure. The reason may be that the amount of methane and the geometric dimensions of pore and crack in coal block are larger if high methane pressure affects them, which will form the methane pressure gradient easily in coal block and make the free methane diffuse outside of coal block and make the absorbed methane in coal block be changed into free methane and diffuse outside of coal block.
(4) Test time when curve of methane diffusion speed enters the third phase is extended gradually but the last trend value of methane diffusion speed is similar although the methane pressure is different. The reason may be that the methane source in the third phase of test curve mainly depends on desorbed methane from coal block; the amount of desorbed methane and free methane in coal block is larger when the methane pressure is increased, which makes the time needed by test extended. After the test enters into the third phase, the internal and external environment where the coal block lies are similar to each other; the influence on methane desorbed properties caused by initial methane pressure is not obvious, especially entering into the stage of residual methane desorbing, so that the law is shown in the test curve.
(5) Test time when the methane diffusion speed is shown in significant value is basically the same under the condition of used sensors in this paper with the increase of methane pressure, but the reason may be the influence of sensors accuracy.
(6) Properties of the methane diffusion speed curve of coal block under triaxial compressive stress can be expressed by the following equation regardless of how to change the initial methane pressure, whose fitting accuracy is larger than 0.9:
  (1) $$\begin{array}{c} v=\left\{\begin{array}{cc} a_{1}\cdot t+b_{1} & \text{the first stage}\\ \frac{a_{2}}{c_{2}\cdot t}+b_{2} & \text{the second stage}\\ a_{3}\cdot t+b_{3} & \text{the third stage}\\ 0 & \text{the fourth stage.} \end{array}\right. \end{array}$$

The influences caused by methane pressure only are shown in the difference of fitting parameters of the above equations.

## 4. Conclusions

The main conclusions can be obtained according to the above tests and analysis as follows.

1. Four-stage properties are very obvious in methane diffusion speed of coal block under triaxial compressive stress, including first is sharply reduce stage, second is hyperbolic reduce stage, third is close to a fixed value stage, fourth stage is 0.
2. There is a special point in test curve of methane diffusion speed of coal block under triaxial compressive stress making the reduction rate of methane diffusion speed sharply decreased in a short time.
3. There is no obviously influences on curve of methane diffusion speed caused by methane pressure, and influences only be shown in size of methane diffusion speed obvious.
4. Equation that properties of the methane diffusion speed curve of coal block under triaxial compressive stress can be expressed was obtained regardless of how to change the initial methane pressure.

## Figures and Tables

**Figure 1:** Thermo-fluid-solid coupling with triaxial servocontrolled seepage equipment of methane-containing coal.

**Figure 2:** Test samples.

**Figure 3:** Characteristic curve of methane diffusion speed (methane pressure is 1.0 MPa).

**Figure 4:** Influences of methane diffusion properties caused by methane pressure.
